# Cytotoxicity and Antibacterial Activity of Mineral Trioxide Aggregate Cement with Radiopacity Introduced by ZrO_2_

**DOI:** 10.1155/2022/9574245

**Published:** 2022-09-06

**Authors:** Lidia Ciołek, Zbigniew Jaegermann, Ewa Zaczyńska, Anna Czarny, Monika Biernat, Arkadiusz Gąsiński, Agnieszka Jastrzębska, Michał Gloc, Andrzej Olszyna

**Affiliations:** ^1^Łukasiewicz Research Network-Institute of Ceramics and Building Materials, Ceramic and Concrete Division in Warsaw, Biomaterials Research Group, Cementowa 8, 31-983 Kraków, Poland; ^2^Polish Academy of Sciences, Institute of Immunology and Experimental Therapy, 12 Rudolf Weigl Street, 53-114 Wroclaw, Poland; ^3^Łukasiewicz Research Network-Institute of Ceramics and Building Materials, Ceramic and Concrete Division in Warsaw, Ceramic Technology Research Group, Cementowa 8, 31-983 Kraków, Poland; ^4^Warsaw University of Technology, Faculty of Materials Science and Engineering, Wołoska 141, 02-507 Warsaw, Poland

## Abstract

The article presents the results of *in vitro* studies on cytotoxicity and antibacterial activity of new MTA-type cements, developed on the basis of the sintered tricalcium silicate enriched with ZnO, along with an agent introducing the radiopacity in the form of ZrO_2_. The new materials have been developed to ensure that their physical and chemical properties are suited for endodontic applications. The cements were evaluated via characterisation of setting time, compressive strength, as well as translucency on X-ray images, and bioactivity in the simulated body fluid (SBF). The *μ*CT was used to test the influence of the ZrO_2_ grains in the powder component on the microstructure of the produced cement. Then, the cytotoxic action of the cements was evaluated by applying a reference L-929 cell line. The conditions of the culture upon contact with the tested materials or with extracts from the cements were assessed using image analysis or an MTT colorimetric assay. Two strains of streptococci, *Streptococcus mutans* and *Streptococcus sanguinis,* were used to study the antibacterial activity of the tested cements with ZrO_2_ acting as the agent introducing the radiopacity. The new cements are characterised by appropriate properties as far as retrograde root canal filling is concerned.

## 1. Introduction

For many years, MTA (Mineral Trioxide Aggregate) type preparations, whose chemical composition is based on tricalcium silicate 3CaO•SiO_2_, have been considered to be preferable materials for retrograde root canal filling [1, 2]. The constitution of mineral trioxide aggregate was described by Camilleri et al. [3]. The authors showed that MTA is composed primarily of tricalcium (3CaO∙SiO_2_) and dicalcium silicate (2CaO∙SiO_2_), which upon hydration produce a silicate hydrate gel (C-S-H phase) and calcium hydroxide (Ca(OH)_2_, portlandite), thus rendering it biocompatible. Retrograde root canal filling proves essential, e.g., in the case of root wall perforation while preparing a post and core crown. If the damage is extensive or there is a risk of shifting the closing material, the perforation cannot be filled in from the side of the canal. In this case, it is essential to close the perforation from the external side, with the damaged site being surgically uncovered. In the course of this therapy, it is recommended to use materials that interact with the pulp or the dentin and maintain tissue viability in order to fill in the lost part of the tooth [4–6]. Current approaches to treating dental pulp suggest selecting therapeutic methods that enable leaving an entirely or partially healthy and vital pulp. Specialists prefer therapeutic methods based on materials supporting the defence and regenerative capabilities of the pulp, which lead to its healing [7, 8]. MTA-type materials are used clinically for their bioactivity and are seen as the most suitable instruments for sealing perforation [9–11]. As presented [12] by Taddei et al., the bioactive behavior of calcium silicate materials may be positively influenced by the presence of phosphorus, which acts as a nucleation agent to accelerate the kinetics of apatite formation. It was also found that the biomineralization process has a positive effect on the push-out strength of cements, especially from the MTA group [13]. This thesis is confirmed by the results of the *in vivo* research presented by Reston et al. [14], whose aim was to study the morphology and location of hard tissues barriers in contact with the ProRoot MTA material. The tissue biocompatibility of MTA-type materials results mainly from their chemical composition [2, 15, 16]. Numerous studies have shown that the MTA stimulates alkaline phosphatase expression, which plays a crucial role in cementogenesis [17, 18]. Cement formation on the surface of the damaged root is an essential condition for the tight sealing of the perforation and regeneration of the damaged tissue. Furthermore, the MTA-type materials are known for their hydraulic character, therefore, they may be used in humid environments, without compromising the quality after setting. The disadvantage of using these types of materials is associated with a relatively long setting time and low compressive strength [19]. Another important feature characterising MTA-type materials is associated with producing calcium hydroxide during the setting reaction, hence the resulting alkaline environment reduces the risk of infection [20]. The presence of certain elements in the composition of the material may also ensure protection against infections. The influence of Ag + ions on microorganisms is explained and documented [21, 22]; however, bactericidal properties have also been reported in the case of other metal ions, such as zinc, copper, gold, and cerium [23–28]. Much attention has been paid to zinc nanoparticles and its biological use due to their compatibility, as well as their unique thermal and optical properties [29–31]. As far as the human organism is concerned, the advantages of zinc have been considered universal, since Zn2+ plays an important role, especially within the immune system. Zinc ions also play a crucial role in metabolic processes, as they are components or activators for many enzymes [32, 33] and have antibacterial properties [24].

MTA-type cements for applications in endodontics should be set in a humid environment, adhere tightly to dental tissues, maintain constant volume, are easy to use, and provide a clear and visible contrast on X-ray images. After application, the demonstrated radiopacity allows these materials to be distinguished from neighbouring anatomical structures. In 1979, Eliasson and Haasken [34] established a comparative reference by using the values of measured optical density and proposed the method of calculating the equivalent thickness of aluminium plates. Most frequently, the radiopacity is introduced by adding gold or silver powder, along with barium sulphate, zinc oxide, or bismuth oxide. Zirconium oxide may be another agent that introduces radiopacity [35]. Cements containing bismuth oxide reveal the inclusion of Bi^3+^ ions into the structure of calcium silicates [36], as well as their leaching from the cement [37]. Clinical observations show that even a slight amount of these ions reveal a certain toxicity and pose a negative influence on the growth of dental cells [38], which may even lead to their necrosis [39]. Long-term clinical observations focusing on MTA cements available in the market indicate the occurrence of discolorations within the surrounding tissues of the dental structure [40], which poses a considerable aesthetic problem for patients.

The overall goal of our research was to develop an MTA-type endodontic cement based on sintered ZnO enriched tricalcium silicate with ZrO_2_ as a radiopacity agent. The aim of the presented work was to determine the level of cytotoxicity and bactericidal activity of the cement with the proposed new chemical composition.

## 2. Materials and Methods

### 2.1. Materials

MK.056/001 (SKSM) silica flour, calcium carbonate (analytical grade) (POCh), calcium hydroxide (analytical grade) (Merck), zinc oxide (analytical grade) (POCh), and aluminium oxide (analytical grade) (POCh) were used to prepare the sintered powder. Zirconium oxide (IV) (analytical grade) (Merck) have been used in the powder component of these cements to introduce the radiopacity.

For *in vitro* studies, the following reagents were used: foetal calf serum (FCS), RPMI-1640 products were purchased from Biowest (Nuaillé, France). L-glutamine, penicillin and streptomycin solution, MTT (3-[4,5-dimethylthiazol-2-yl]-2,5-diphenyltetrazolium bromide), DMF (dimethylformamide), SDS, and trypan blue were obtained from Sigma-Aldrich (Munich, Germany), and the growth media such as Brain-Heart broth (BHI), TSA medium (Trypton-Soy-Agar) with 5% blood purchased from BTL Ltd., (Enzymes and Peptones Department in BTL Ltd., Łódź, Poland), and 0.9% NaCl solution (Institute of Immunology and Experimental Therapy of the Polish Academy of Sciences, Wrocław, Poland).

### 2.2. Sintered Powders Preparation Procedure

A mixture corresponding to the composition of the tricalcium phosphate in the CaO-SiO_2_-Al_2_O_3_-ZnO system was designed. Due to the belief that changes in the reactivity of various phases of 3CaO•SiO_2_ in relation to water are mainly associated with structural defects [41], 0.3wt.% of the SiO_2_ within the chemical composition of the mixture was replaced with the same amount of aluminium oxide and 1wt.% of CaO was replaced with ZnO. The mixture was sintered to prepare the powder component for the MTA-type cement. The raw materials had the following forms: calcium carbonate with the calcite structure (CaCO_3_), calcium hydroxide with the portlandite structure (Ca(OH)_2._), silicon dioxide with the quartz structure (SiO_2_), zinc oxide with the zincite structure (ZnO), and aluminium oxide with the corundum structure (Al_2_O_3_). A mixture was homogenised in a special porcelain ball grinder. The degree of homogenisation was confirmed with X-ray diffraction tests by comparison of four samples taken from different places. Then, the mixture was placed in a ceramic crucible, sintered at a temperature reaching 1480°C/6h in an electric furnace and milled. The grinding and sintering were repeated three times to maximize the reaction between CaO and SiO_2_. As the synthesis of tricalcium silicate took part in the solid phase, after each curing the input was ground in the ball mill for 1 h with 28 mm alumina grinders, in order to obtain better homogenisation. After the third sintering, the product was ground in a rotary-vibratory mill for 1 h with 6 mm zirconia grinders. In total, three syntheses were carried out, as a result of which three batches of sintered powders were obtained (A, B, and C). Each batch of powder was tested to identify the phase composition and granulation.

### 2.3. Characteristics and Properties of the Produced Cement

#### 2.3.1. XRD of the Powders

The analysis of the mineral composition of samples from the sintered powders was performed with the X-ray diffraction method in the Bragg-Brentano geometry using the Bruker-AXS D8 DAVINCI diffractometer, equipped with a copper anode lamp. The diffractograms were registered within angles ranging from 5 to 120° 2*θ* (Cu K*α*), the time measurement interval was 0.01° and the measuring time was 2 s/interval. The optical system of the diffractometer included a 0.3° divergence slit, a 1.5° antiscatter slit, a 2.5° Soller slit, a Ni filter, and the LynxEye strip detector with the field of vision equal to 2.94°. Phase identification was performed by comparing the registered diffractograms with standards registered in the ICDD PDF-2 and PDF-4+ 2016 base with the use of the DIFFRACplus EVA-SEARCH programme.

The results of the standardless analysis were obtained on the EDXRF Epsilon 4 spectrometer from Malvern Panalytical. Powder samples within the scope of C-Am were submitted for elemental analysis. Tests were performed on the device acting on the basis of energy dispersion (EDXRF) equipped with an X-ray lamp with a 15 W Rh anode and a 50 kV and 3 mA generator, a set of 6 measuring filters, and a high resolution SDD semiconductor detector cooled according to the Peltier effect.

#### 2.3.2. Particle Size Analysis of the Ingredients in the Powder Component

The particle size analysis was performed with a laser analyser from Malvern Instruments Mastersizer 2000 using the low angle laser light scattering method (LALLS). The device enables the analysis of a wide range of grains, from 0.1 *µ*m to 2000 *µ*m, with a possible error of 0.5%. Due to the hydrolytic activity of the sintered powders, the samples were dispersed in isopropyl alcohol. Apart from the complete particle size distribution, the analysis report was generated by the Mastersizer 2000 Ver. 5.60 software.

#### 2.3.3. FTIR of ZrO_2_ Used as the Agent Providing the Radiopacity

FTIR analysis of ZrO_2_ was performed with the use of a FTIR TENSOR27 Bruker spectrometer. The measurement was carried out in transmission mode (samples in the form of KBr pellets), in the wavenumber range of 400–4000 cm^−1^, number of scans 64/64, resolution 4 cm^−1^.

#### 2.3.4. Setting Time and Kneading Capacity of the Cements

The setting time for the cements was determined according to standard ISO 9917–1 [42] at a temperature of 37 ± 1°C with a penetrometer weighing 160 ± 5 g with a flat-tip needle with a diameter of *ø* = 1 mm. After filling a cylinder-shaped mould (*d* = 10 mm and *h* = 5 mm) with the material in a plastic condition, the test was performed by lowering the penetrometer tip vertically onto the surface of the material and leaving it there for 5 s. The needle of the penetrometer was lowered in 10-second intervals until it stopped leaving circular indentations in the material, visible after 2× magnification. The setting time was described as the time between the end of the mixing process and the moment when the needle stopped leaving circular traces on the surface of the cement. The kneading capacity of the cements, namely, the capacity to form a homogeneous mixture from the powder component and liquid, was evaluated based on a four-point scale: 1^*∗*^ – very easy to knead, 2^*∗*^ – requires longer kneading, 3^*∗*^ – difficult to knead, 4^*∗*^ – impossible to knead.

#### 2.3.5. Compressive Strength

The compressive strength was determined according to standard ISO 9917–1 [42] with the use of the LR 10R testing machine from Lloyd Instruments with a measurement range between 2 and 9500 N, and a head feed speed equal to 0.75 mm/min. The mixed cements were placed, with a slight surplus, in stainless steel cylinder-shaped moulds (*ø* = 4 mm and *h* = 6 mm). At least 6 samples were prepared for each series of the tested cement. After 1 h, the samples were ground, taken out of the moulds, immersed in water, and stored for 23 h in a dryer at a constant temperature of 37 ± 1°C. The results obtained were presented as mean values.

#### 2.3.6. Evaluation of the Radiopacity

Samples for testing were prepared according to standard ISO 9917–1 [42] in the form of circles with a diameter of 10 mm and *h* = 2 or 3 mm, along with templates made of Al in the form of cuboids with a side of 10 mm and *h* = 5 mm, 6 mm, 7 mm and 8 mm. The samples, along with the templates, were placed on a radiological FOMA DENTIX film used to take 30 mm × 40 mm occlusal photos and having *E* speed (Kodak) and they were irradiated with X-rays with the GENDEX DC DENS extraoral radiograph with the exposure conditions maintained: 65 kV and 7.5 mA. The distance between the tube of the device and the surface of the film was 2 cm. After exposure, the film was processed in an automatic X-ray imager, which provided radiological images with various degrees of translucency. The digital radiological images were used to visually compare the translucency degree of the cement circles and the Al template plates.

With this method, the higher radiopacity on the film provides a more translucent image after processing. Materials appropriate for endodontic fillings in the form of 1 mm thick matrices should have a radiopacity compared with a 3 mm thick Al plate, because the Al equivalent assumed for the 1 mm thick dentin layer was 1 mm, and for the 1 mm enamel layer it was 2.1 mm.

#### 2.3.7. Determination of As and Pb Content in the Set Cement

The arsenic content was determined with a spectrophotometric method using the Spekol 11 spectrophotometer from the Carl Zeiss Jena company. The determination was based on absorbing arsine and measuring the absorbance at a wavelength of 540 nm.

The lead content was determined with flame atomic absorption spectrometry (FAAS), using the SpektrAA 200 spectrophotometer from the Varian company. The measurement was performed at a wavelength of 217 nm. In order to prepare the samples for these tests according to standard ISO 9917–1 [42], appropriate amounts of the powder and liquid were mixed for each of the cements to obtain at least 4 g of the cement. The cements in a plastic condition were placed in the polyethylene foil and then sealed tightly. The cements were then flattened and pressed with fingers to form thin circles. Then, these circles were placed in the incubator for 24 h at 37 ± 1°C. After 24 h, the circles were crushed into fine powder in the agate mortar. The obtained powder was sieved through a sieve with a mesh size of 40 *µ*m.

#### 2.3.8. Bioactivity in the SBF Solution

In order to determine the *in vitro* bioactivity of the produced MTA-type cements, the effect was evaluated with the use of a simulated body fluid (SBF). Therefore, 5 cement circles were placed in tightly sealed glass vessels and then 65 ml of the SBF solution was introduced into each of these vessels. The vessels were placed in a dryer at a constant temperature of 37°C for a period of up to 28 days. The ionic composition of the SBF solution is presented in Table 1.

Microscopic observations were performed using a field emission scanning electron microscope (Nova NanoSEM 200, FEI). Imaging of nonsputtered samples was conducted in low vacuum conditions using a vCD detector at 10 kV accelerating voltage. Nonmodel chemical analysis involving superficial effects after incubation of cements in a Simulated Body Fluid and in low vacuum conditions was performed using EDS detector, SDD Apollo *X* model, and EDAX.

#### 2.3.9. Analysis of the *μ*CT of the Set Cement

The measurements were performed on the SkyScan 1172 X-ray microtomograph. The following parameters were applied: 100 kV, 100 *μ*A, 600 X-ray projections, and an exposure time of 2.5 s.

#### 2.3.10. Cytotoxicity Test

The *in vitro* cytotoxicity of the biomaterial was tested by direct and indirect contact with the monolayer cell culture L-929 fibroblasts (American Type Culture Collection Certified Cell Line‐ATCC CCL1). The mouse fibroblastlike cell line was maintained in an RPMI-1640 medium at 2 × 10^5^ cells/mL supplemented with 10% calf serum (c.s.), antibiotics (100 U/ml of penicillin, 100 *µ*g/ml of streptomycin), and 2 mM·L‐glutamine. The cells were maintained at 37°C in a humidified incubator with 5% CO_2_ for 24 h, until a monolayer, with a confluence greater than 80%, was obtained. They were detached using a mixture of 0.125% trypsin and 0.025% ethylenediaminetetraacetic acid (EDTA). Before starting the tests, the cements were exposed to a UV lamp for 45 min at room temperature. Cell growth, morphology, and viability (Trypan Blue Staining) were determined using image analysis methods. The level of toxicity was defined according to the requirements presented in EN ISO 10993–5:2009.

### 2.4. Direct Contact Cytotoxicity Test

The *in vitro* cytotoxicity test of the cement was carried out by direct contact with the monolayer cell culture L929 fibroblasts. The L929 cells were seeded in 24-well plates (Costar) with 1000 *µ*L per well (at the density of 1 × 105 cells/mL). After 24 h, the supernatant was removed and 1 ml of an RPMI-1640 medium with 2% calf serum was poured in. The cell culture area was covered with the cement and incubated for 24, 48, and 72 h at 37°C in an atmosphere of 5% CO_2_ in the air.

### 2.5. Indirect Contact Cytotoxicity Test

In the indirect methods, the monolayer cell culture L929 fibroblasts were covered with 1000 *µ*L of extract from the cements. The extract from the cements was prepared using an RPMI-1640 medium without calf serum, supplemented with 100 U/ml of penicillin, 100 *µ*g/ml of streptomycin, and 2 mM of L-glutamine. The L-929 cell culture with extracts from materials was incubated for 24, 48, and 72 h at 37°C in the atmosphere of 5% CO_2_ in the air.

### 2.6. Trypan Blue Staining for Cell Viability

The conditions of cultures coming into contact with the tested materials (direct method) or with extracts from these materials (indirect methods) were assessed using image analysis. Cell growth, cell morphology, and cell viability (Trypan Blue Staining) were used as parameters to determine the cytotoxicity of the cement samples. The trypan blue exclusion method was used for cell viability, where 100 *µ*L of cell suspension (2 × 10^6^ cell/mL) was incubated with 100 *µ*L of 0.4% trypan blue. The viability of the cells in a Bürker chamber was then measured. Dead cells were labelled with navy blue, and living cells remained unstained. The morphology of the cells was assessed using an inverted microscope at 400× magnification, according to the criteria set out in Table 2. Each test using cement in the direct method or its eluate in the indirect method was performed three times and representative test results were presented.

### 2.7. Colorimetric MTT Assay for Cell Growth

The MTT colorimetric assay [43] was used to establish the viability of cells. Briefly, 25 *μ*l of the MTT (5 mg/ml) stock solution was added per well at the end of the cell incubation period and the plates were incubated for an additional 3 h in a cell culture incubator. Then, 100 *μ*l of the extraction buffer (20% SDS with 50% DMF, pH 4.7) was added. After overnight incubation, the OD was measured at 550 nm with the reference wavelength of 630 nm in a Dynatech 5000 spectrophotometer.

#### 2.7.1. Study of Antibacterial Activity

The following microorganisms were used for *in vitro* studies: *Streptococcus mutans* ATCC 25175 derived from tooth decay and *Streptococcus sanguinis ATCC BAA-1455* isolated from plaque. Bacterial strains were purchased from the American Collection of Microorganisms (ATCC). The studies were based on the dilution method. The preculture of streptococcal test strains, *S. mutans* and *S. sanguinis,* was incubated in a brain heart infusion broth at 37°C for 18–20 h in an anaerobic atmosphere. 1 ml of a 10× diluted bacterial culture was applied to the wells of a 24-well plate, and then sterile test material was placed. After 24 h, 48 h, and 7 days of incubation, 100 *µ*l of the bacterial culture was taken, diluted with 0.9% NaCl and plated (100 *µ*l) onto tryptic-soy agar plates with 5% blood. The plates were incubated overnight at 37°C in an anaerobic atmosphere and the colony forming units were counted (CFU/ml). Microorganisms in broth cultures, free from the tested materials, constituted the control group.

### 2.8. Statistical Analysis

The results are presented as mean values ± SD (standard deviation). The Brown-Forsythe test was used to examine the homogeneity of variance between groups. When the variance was homogeneous, the statistical analysis was performed by analysis of variance (ANOVA), which was then followed by posthoc comparisons with Tukey's test to estimate the significance of the difference between groups. Nonparametric data were evaluated with the Kruskal–Wallis analysis of variance. The significance was determined at *P* < 0.05. The statistical analysis was performed using STATISTICA 7.0 for Windows.

## 3. Results and Discussion

### 3.1. Characteristics of the Sintered Powder

After being ground and subjected to the granulation evaluation process on a 50 *µ*m sieve, the tricalcium silicate sinters produced were characterised by granulation presented in Table 3.

The characteristic value of granulation relating to 50% of the volume in the population of particles did not exceed 7.93 *µ*m for sintered powder A, 7.98 *µ*m for sintered powder B, and 7.03 *µ*m for sintered powder C.

### 3.2. Results of the XRD Analysis and (EDXRF)

Three samples were collected from each batch of the product and then tested with the XRD method to verify the homogeneity of the material. Alite, tricalcium silicate (3CaO∙SiO_2_) was found to be the main phase (Figure 1). In addition, the presence of dicalcium silicate, larnite (2CaO∙SiO2) was also observed. The diffractograms obtained indicate that the synthesis method used, based on multiple curing and grinding processes applied to the properly prepared raw material components, allows the production of homogeneous and repetitive sintered powder. The XRF quantitative analysis was performed for the sample marked with the symbol B. The analysis focusing on the chemical composition of the sintered powder took into consideration the additional participation of ZrO_2_ coming from zirconia grinders. The ground sintered powder (ED-XRF) contained 71.23% wt. of CaO; 26.59% wt. of SiO_2_; 1.31% wt. of Al_2_O_3_, 0.75% wt. of ZnO, and additionally 0.12% wt. of ZrO_2_. The excess of Al_2_O_3_ and ZrO_2_ with respect to initial composition results from using of alumina and zirconia grinders during milling.

The sintered powder B constituted the basis for developing the composition of the powder component of the MTA cement. Freshly prepared aqueous CaCl_2_ solution with a concentration equal to 10% wt. or 15% wt. was used as the liquid. During this experiment, the ratio between the powder component and the liquid was 3.0 g/1.0 ml and 3.6 g/1.0 ml. The following parameters were determined for the cements prepared in the above-mentioned manner: kneading capacity, setting time, and compressive strength. All the cements were characterised by incredibly high kneading capacity. The impact of powder/liquid proportions and CaCl_2_ concentration on the setting time, compressive strength, and kneading capacity of the cements was shown in Table 4.

The cement obtained from 3.6 g powder and 1.0 ml liquid (15% wt. CaCl_2_ solution) was characterised by a shorter final setting time and considerably higher compressive strength. The cement kneaded in the same powder/liquid proportion (10% wt. CaCl_2_ solution) also revealed a high compressive strength, however, the final setting time was longer in this case. The cements were kneaded with 3.0 g powder per 1.0 ml of 15% weight and 10% wt. CaCl_2_ solution showed compressive strengths of 94.0 MPa, and 86.2 MPa, respectively, and the final setting time of 48 min and longer than 60 min. The obtained final setting times for the developed cements are comparable with other cements of the MTA type, which are described in publication [44]. Taking into consideration the results and the need to include the radiopacity introducing agent in the powder component, the 3.6 g of powder/1.0 ml of 15% wt. CaCl_2_ solution proportion was selected for further tests. With the selected proportion and concentration of the liquid for kneading, the shortest setting time for cement was obtained, along with the highest compressive strength. Then, for the selected powder/liquid proportion and the CaCl_2_ solution concentration, the performance of the cements was evaluated for all the sintered powders and the impact of the granulation of the powder component was verified. The results obtained differed slightly. With sintered powder A, a cement with the longest setting time and the smallest compressive strength was obtained (Table 5). This result may prove that the grains of sintered powder B and C, characterised by a lower Dv (0.1) shorten the setting time due to a larger specific surface, where the setting reactions take place. It was also observed that the faster setting cements revealed a greater compressive strength. The ease in creating the firm texture of the cement by faster setting reactions of smaller grains should facilitate the work of clinicians during application.

The sintered powder B and ZrO_2_ were applied to prepare the powder component of the cement. As the radiopacity agent, ZrO_2_ with the Dv (0.1), Dv (0.5), and Dv (0.9) grain sizes of 6.49 *µ*m, 14.24 *µ*m, and 25.90 *µ*m, respectively, was used. The characteristic value of the granulation Dv (0.1) and Dv (0.5) in the case of the zircon oxide used was higher, and the Dv (0.9) was lower than that of the sintered powder (Table 3). The components of the powder were mixed in a rotary-vibratory mill without grinders for 30 min. The participation of ZrO_2_ in the prepared powder components were of 0, 10, 20, 25, 30, and 40% wt. Increasing the participation of the radiopacity agent in all the tested materials resulted in prolonging the setting time. As we showed in our previous article [45] with a 10% wt. addition of ZrO_2_ in the powder component, a slight increase in the compressive strength was observed when compared with the compressive strength of the cement without the addition of ZrO_2_. According to Coleman [46], the zircon oxide grains ranging in size between 0.2 and 5.0 *µ*m, which do not participate in the cement setting reactions, can constitute a nucleation site for precipitation and growth of early products of its hydration reaction. Therefore, one may conclude that the observed increase in compressive strength might have been related with the presence of very small grains of ZrO_2_. However, as we showed previously, with a higher than 10% wt. share of ZrO_2_ in the powder component, being an inert agent as far [45] as the cement setting reaction is concerned, decreased compressive strength was observed. Regardless of the amount of ZrO_2_ powder introduced, the workability of the cements did not deteriorate. The radiopacity of cements was evaluated by comparing the degree of their translucency in X-ray images with the translucency of aluminium (Al) equivalents. A cement sample containing 10 wt.%. ZrO_2_ absorbs X-ray radiation just like the Al standard with a thickness of 5 mm, i.e., its translucency is equivalent to 3 mm of dentin with a 1 mm layer of enamel. The obtained result can be considered comparable to that presented by Coleman [46] for Biodentine (1.5 mm Al for a sample with a thickness of 1 mm). At 20 wt.% ZrO_2_ in the cement, the obtained degree of translucency is comparable to the Al standard with a thickness of 7 mm. The optimum contrast on X-ray images was observed in the case of the cement containing 25% wt. ZrO_2_ weight in the powder component. With this participation of ZrO_2_, the translucency of the cement was equivalent to the 8 mm thick template Al plate, which corresponds to 6 mm of dentin with a 1 mm enamel layer. The obtained result is adequate for endodontic sealing material which should present radiopacity corresponding to at least 3 mm Al which was reported by Borges [47]. The setting time for this cement exceeded 60 min, and the compressive strength reached 97.5 ± 9.3 MPa. The setting time for clinically applied Biodentine and ProRoot MTA cements, as stated by Kaup [48], is 85.66 min and 228.33 min respectively. However, it is worth mentioning that tests were conducted using a smaller diameter needle in the penetrometer and a greater load than the recommended one.

Samples of the cement with 25% wt. of ZrO_2_ (with the optimum contrast on X-ray) were prepared for biological tests. The first attempt to perform *in vitro* tests was unsuccessful because the cement samples with the radiopacity agent changed the morphology of the cement surface, which resulted in a toxic effect on cells. The above-given observation was made after the addition of the ZrO_2_ powder which is known as biocompatible. Hence we made the assumption that the ZrO_2_ powder we used may contain an additional organic substance, derived from the production process. In order to confirm these assumptions, an FTIR test was performed.

On the FTIR spectra (Figure 2) the main absorption band appeared at 746, 577, and 523 cm^−1^ which is characteristic for stretching vibrations of Zr-O in ZrO_2_. In addition, the weak absorption bands were identified in the range of 1600–1700 cm^−1^ and in the range of 2850–2950 cm^−1^, corresponding to bending and stretching vibrations of C–H in CH_2_ groups probably derived from the organic substance. In order to get rid of the organic phase that contaminates the ZrO_2_, thermal treatment (600°C) was carried out. The treatment was carried out for two different samples. In the sample marked as (C + ZrO_2_)/600°C the sintered powder was first mixed with ZrO_2_ and the whole mass was then submitted to thermal processing at 600°C. In the second sample, marked as C+(ZrO_2_/600°C), the ZrO_2_ was first submitted to thermal processing and then combined with the sintered powder. The samples of the cement for cytotoxicity tests and antibacterial activity tests were prepared by mixing the powder component with the kneading liquid in the 3.6 g/ml proportion. “C” marked cement with no addition of ZrO_2_ was the reference sample.

### 3.3. Determination of As and Pb Content in the Set Cement

Determination of cement contamination with arsenic and lead is important due to the toxic effects of these elements, which may be present in the cement composition from the raw materials or during the manufacturing process. To confirm the chemical composition's safety of the developed material, the content of As and Pb soluble in dilute hydrochloric acid was marked in the set cement prepared on the basis of sintered powder B with an addition of 25% wt. of ZrO_2_ and the liquid (15% wt. CaCl_2_ solution). As far as the tested material is concerned, the arsenic and lead content were below the limit of quantification marked with the use of this method.

### 3.4. The Results of the *μ*CT Analysis

Two cements prepared on the basis of sintered powder B, differing as far as the composition of their powder component is concerned (Table 6), underwent the *µ*CT analysis (Figure 3).

Sample 1: cement from only the sintered powder kneaded with 3.6 g of powder/1.0 ml 15% wt. CaCl_2_. Sample 2: cement (B25Zr) where 25% wt. ZrO_2_ was added to the powder component instead of the sintered powder B and then kneaded in an identical proportion. During the three-dimensional visualisation, the participation of pores in sample 1 was evaluated to be 0.8%, whereas the average size of pores was 29.9 ± 12.3 *μ*m. In sample 2, the participation of pores was significantly lower and reached 0.1%, while the average size of pores was 23.8 ± 13.8 *μ*m. The identified differences can result mainly from the sintered powder filling intergranular spaces with considerably smaller ZrO_2_ grains present in sample 2. The density of the structure of cement (B25Zr) had a positive impact on the improvement in the radiopacity.

### 3.5. SEM-EDS Bioactivity

In the case of the B25Zr cement sample before incubation in SBF, signals from O, Ca, and Zr were present in the cement (Figure 4(a)). The different intensity of the signal from Zr was related to the homogeneity of the mixture. After cement incubation in SBF, the signal intensity from O, Mg, and Si changed, which was associated with the creation of spherical structures on the surface of the cement (Figure 4(b)). The presence of P was not identified in the SEM-EDS analysis, although the 10 kV excitation energy used was adequate to identify this element. The calcium ions released from the MTA-type material are essential for the migration, differentiation, and proliferation of hard tissue producing cells, e.g., hydroxyapatite according to the mechanism described in the article by Tanomaru et al. [49] where a comparison of MTA and tantalum oxide NeoMTA containing materials is presented. Early nucleation of hydroxyapatite crystals, may be improved by the presence of fluoride in the composition of the material. As presented by Gandolfi et al. [50] fluoride-doped calcium silicate cements are better able to form apatite (bioactivity) and are more reactive than conventional calcium silicate cements. However, the reactivity of the cement presented in this paper is mainly related to the structural defects of the sintered powder [41]. The calcium needed to create a hydroxyapatite layer, which proves the bioactivity of the tested material, was provided by the chemical composition of the MTA cement powder, and phosphorus as well as magnesium were in the simulated body fluid (SBF) solution.

### 3.6. Cytotoxicity Assay

#### 3.6.1. Estimation of the Cytotoxicity of Tested Compounds on the L-929 Reference Cell Line

The cytotoxic action of the obtained cements was evaluated by applying a reference cell line. The conditions of cultures in contact with tested materials (direct method) or with extracts from the cements (indirect method) were assessed using image analysis or the colorimetric MTT method. The level of cytotoxicity of the cements was determined by measuring the growth of the fibroblast mouse L-929 cell line for 24, 48, and 72 h at 37°C.

#### 3.6.2. Trypan Blue Staining

Image analysis using Trypan Blue Staining was utilised to determine the level of cell viability after the period of incubation. The results are presented in Table 7. The highest decrease in cell viability was observed after 72 h of indirect contact with C+(ZrO_2_/600°C) cement (44.8%). According to the 4-point scale presented in Table 2, this level of changes in cell cultures corresponds to the 2nd degree of toxicity. Therefore, cement C+(ZrO_2_/600°C) can be considered a mildly toxic material *in vitro*. A much better effect was obtained for (C + ZrO_2_)/600°C cement, as after 72 h there was a decrease of only 1.7%, which according to accepted criteria can be considered a slightly toxic material *in vitro.*

#### 3.6.3. MTT Assay

In the MTT colorimetric assay, the optical density (OD) was measured and the cellular metabolic activity of mouse fibroblast cell line L-929 in the presence of the cements and their eluates was determined. The L-929 mouse fibroblasts after direct contact with all the considered materials demonstrated almost a stable viability level and the statistical analysis showed no significant difference after 24, 48, and 72 h of direct contact (Figure 5). However, based on the results of the OD studies, it was concluded that C+(ZrO_2_/600°C) had a statistically significant effect on the cells by slowing down their metabolism after 72 h in indirect contact (Figure 5(c)). The best result in the MTT assay was obtained for the (C + ZrO_2_)/600°C cement, similarly to the Trypan Blue Staining method. The results obtained emphasize the impact of the powder component preparing method. Despite the same sintered powder/ZrO_2_ ratio in the tested samples, the C + cement (ZrO_2_/600°C) had a higher effect on cell metabolism than in the case of (C + ZrO_2_)/600°C. The obtained results may indicate that the undesirable organic substance was better removed during the applied thermal treatment from the sample in which the ZrO_2_ grains and the sintered powder were mixed before annealing.

Proliferation and migration of cells is a key event in tissue repair and regeneration [2]. In an article by A. L. Gomes-Cornelio 2017 [51] the results of MTT tests for other MTA-type materials are presented. In the presented results the material containing ZrO_2_ as well as MTA Plus and Biodentine showed higher viability and proliferation rates compared to the control.

#### 3.6.4. Antibacterial Properties

Two strains of streptococci, *Streptococcus mutans* and *Streptococcus sanguinis,* often found on the surface of teeth, were used to study the antibacterial activity of the tested cements enriched with ZrO_2_. The bacteria were incubated in the presence of the cement samples for 24 h, 48 h, and 7 days, plated on the appropriate medium, and colonies were counted after overnight incubation. The results of the antibacterial activity of the tested materials against bacterial strains are presented in Figure 6. As shown (Figure 6(a)), after 24 h of bacterial incubation with cements, the number of bacteria of the *Streptococcus mutans* strain was slightly lower when compared with the control (bacterial culture without tested samples). In the case of the *Streptococcus sanguinis* strain, a significant reduction in the number of bacteria, compared to the control, was observed. After 48 h of incubation (Figure 6(b)), the tested cements inhibited the growth of *Streptococcus sanguinis* as well as *Streptococcus mutans*. In the case of *Streptococcus sanguinis*, there was a greater reduction in the number of bacteria, when the strain was grown in the presence of a cement sample C + (ZrO_2_/600^o^C), whereas the count of *Streptococcus mutans* was reduced the most in the presence of a cement sample (C + ZrO_2_)/600^o^ C. As shown (Figure 6(c)), after 7 days of incubation, all tested cements caused a reduction in the number of bacteria of bacteria of both strains, when compared to the control. The presented data show that the tested cements reduced the number of bacteria in comparison with the control. The differences between the antimicrobial activity of the individual cements were minimal. The antibacterial properties of the tested samples depended on the methods of preparing the powder components of cements, as well as on the bacterial strain and the incubation time.

The results of our preliminary studies on the biomaterials indicate a suppressive effect of ZrO_2_ enriched MTA cements on the growth of *Streptococcus mutans* and *Streptococcus sanguinis* in suspension. Silva et al. [52] showed that MTA repair HA cement significantly inhibited *Streptococcus mutans* biofilm formation, however, extracts from this biomaterial did not lower bacterial numbers in suspension. The physicochemical properties of biomaterials affect their antibacterial activity. Metal nanomolecules exhibit antibacterial and even bactericidal activities. The positive charge of ZrO_2_ facilitates the formation of electrostatic bonds with a negatively charged bacterial wall (for example with peptidoglycan) that leads to the accumulation of ZrO_2_ molecules on bacterial surfaces, and in consequence, disturbance in cell membrane permeability, their penetration into bacterial cells and inhibition of important metabolic functions [53]. The diffusion of nanomolecules across bacterial wall depends on their shape and size. Jangra et al. [54] showed that ZrO_2_ molecules of the same area but different shape had different antibacterial activity, i.e., smaller molecules of spherical shape exhibited higher antibacterial activity. ZnO nanomolecules in MTA biomaterial, characterised by antibacterial activity, may also contribute to the reduction of bacteria numbers. It should be also mentioned that other external factors, such as bacteriologic culture media (for example LB bullion) lower the antibacterial effects [55]. The difference in the bacteria numbers between *Streptococcus mutans* and *Streptococcus sanginis*, registered in our study after 24 h incubation in the presence of MTA, could be due to differences in interactions of the strains with the nanomolecules. Ahu et al. [56] demonstrated differences in affinities to orthodontic apparatuses between several strains of S*treptococcus mutans* and *Streptococcus sobrinus*.

## 4. Conclusions

The powder component for the MTA-type cement was produced based on a tricalcium silicate sintered powder enriched with ZnO. ZrO_2_ was used as an agent introducing a radiopacity. With the participation of 25% wt. ZrO_2_ in the powder component, the resulting radiopacity was characterised by a translucency degree corresponding to 6 mm of dentin with a 1 mm layer of enamel, and an appropriate performance was achieved. Both in the direct contact and the indirect contact tests, the lowest toxicity against L929cells was shown by the (C + ZrO_2_)/600°C cement, where thermal processing was applied after including the ZrO_2_ in the powder component. The tests also proved the antibacterial activity of the manufactured cement towards strains of streptococci, namely, *Streptococcus mutans* and *Streptococcus sanguinis*. The addition of ZrO_2_ to biomaterials does not only improve their radiopacity but also enhances the antibacterial activity, that prevents the development of secondary dental decay, frequently being a cause of endodontic procedure failures.

This new proposed composition of the MTA-type cement, produced on the basis of the sintered powder enriched with ZnO and zirconium oxide (IV) is characterised by an appropriate performance and can be considered an endodontic material. However, to consider this cement a safe medical device for retrograde root canal filling, further tests are required, that meet the ISO 10993 standard as well as aim to evaluate its genotoxicity, irritation, and sensitisation effects.

## Figures and Tables

**Figure 1:** XRD patterns of sintered powders A, B, and C along with the identification of marked phases. Producing the MTA-type cement and its characteristics.

**Figure 2:** FTIR spectra of ZrO_2_ were used as the agent providing the radiopacity.

**Figure 3:** Analysis of the *µ*CT of the set cement: (a) Three perpendicular sections: traverse A longitudinal B and sagittal C along with their spatial visualisation D (b) Visualisation of sample pores in a two-dimensional image.

**Figure 4:** SEM images of B25Zr cement and EDS analyses: (a) before incubation in SBF (point 1 - cement surface, point 2 – grain of ZrO_2_); (b) after 28 days of incubation in SBF (point 1 – cement surface).

**Figure 5:** The cytotoxicity effect of tested cements and their eluates after direct and indirect contact on a L-929 cell culture, *in vitro* after incubation for (a) 24 h (b) 48 h, and (c) 72h Cell viability was determined with an MTT colorimetric assay. The results of cytotoxic tests are presented as mean values of optical density (OD) at 550–630 nm ± standard deviation (SD) from three separate experiments are shown; ^*∗*^*P* < 0.05 as compared with control cells.

**Figure 6:** Antibacterial activity of tested cements against *Streptococcus mutans* and *Streptococcus sanguinis* after incubation for (a) 24 h (b) 48 h, and (c) 7 days. This figure shows the number of viable bacteria–CFU/ml.

**Table 1:** Ionic composition of the SBF solution.

	Ion type and concentration (mM/dm^3^)							
	Na^+^	K^+^	Mg^2+^	Ca^2+^	Cl^−^	HCO_3_^−^	HPO_4_^2−^	SO_4_^2−^
SBF	142.0	5.0	1.5	2.5	148.8	4.2	1.0	0.5
Plasma	142.0	5.0	1.5	2.5	103.0	27.0	1.0	0.5

pH of the solution buffered with TRIS and HCl was 7.25.

**Table 2:** Criteria of toxicity effect based on changes in cell morphology according to EN ISO 10993–5:2009.

Grade toxicity	Reactivity	Conditions of all cultures
0	None	Discrete intracytoplasmatic granules, no cell lysis, no reduction of cell growth
1	Slight	Not more than 20% of the cells are round, loosely attached and without intracytoplasmatic granules, or show changes in morphology; occasional lysed cells are present; only slight growth inhibition observable.
2	Mild	Not more than 50% of the cells are round, devoid of intracytoplasmatic granules, no extensive cell lysis; not more than 50% growth inhibition observable.
3	Moderate	Not more than 70% of the cell layers contain rounded cells or are lysed; cell layers not completely destroyed, but more than 50% growth inhibition observable.
4	Severe	Nearly complete or complete destruction of the cell layers.

**Table 3:** Values characteristic for the granular composition of sintered powders A, B, and C.

Symbol of the sintered powder	Characteristic value of the granulation (*µ*m)		
	Dv (0.1)	Dv (0.5)	Dv (0.9)
A	1.05	7.93	25.04
B	0.91	7.98	29.60
C	0.93	7.03	30.70

**Table 4:** Impact of powder/liquid proportions and CaCl_2_ concentration on the setting time, compressive strength, and kneading capacity of the cements, when compared with the reference cement.

Symbol of the sintered powder	Powder/liquid proportion (g/ml)	Type of liquid	Final setting time (min)	Compressive strength (MPa)	Remarks on kneading
B	3.6/1	15% wt. CaCl_2_	27	136.8 ± 9.3	1^*∗*^
		10% wt. CaCl_2_	60	125.0 ± 12.1	1^*∗*^
	3.0/1	15% wt. CaCl_2_	48	94.0 ± 6.8	1^*∗*^
		10% wt. CaCl_2_	>60	86.2 ± 5.6	1^*∗*^

1^*∗*^ – very easy to knead.

**Table 5:** Impact of the sintered powder granulation on the final setting time, compressive strength, and kneading capacity of the cements kneaded with the following proportions: 3.6 g of the sinter/1.0 ml of the 15% CaCl_2_ solution.

Symbol of the sintered powder	Final setting time (min)	Compressive strength (MPa)	Remarks on kneading
A	38	121.5 ± 9.9	1^*∗*^
B	27	136.8 ± 9.3	1^*∗*^
C	30	137.4 ± 9.4	1^*∗*^

1^*∗*^ – very easy to knead.

**Table 6:** Symbols and composition of cements undergoing the *µ*CT test.

Symbol of the cement in *μ*CT tests	Powder component of the cement		Kneading liquid
	Share of sinter B (% wt.)	Share of ZrO_2_ (% wt.)	
Sample 1	100	0	15% wt. CaCl_2_
Sample 2	75	25	15% wt. CaCl_2_

**Table 7:** Percentage of viable L929 cells after the direct and indirect contact with the tested circles, *in vitro.*

Time (h)	Material	Direct contact		Indirect contact	
		Living cells (%)	±SD	Living cells (%)	±SD
24	C	91.0	0.9	97.8	2.1
	(C + ZrO_2_)/600°C	86.7	2.0	92.2	2.7
	C+(ZrO_2_/600°C)	76.9	1.5	80.0	1.4

48	C	90.2	8.1	104	9.9
	(C + ZrO_2_)/600°C	84.7	4.3	99.8	8.5
	C+(ZrO_2_/600°C)	76.8	0.1	93.5	0.9

72	C	82.2	6.8	92.5	8.4
	(C + ZrO_2_)/600°C	81.4	2.0	98.3	8.2
	C+(ZrO_2_/600°C)	86.2	3.3	55.2	5.3

## Data Availability

The data generated during this study are available at ŁUKASIEWICZ Research Network, Institute of Ceramics and Building Materials, Ceramic and Concrete Division in Warsaw, Biomaterials Research Group, Postępu 9, Warsaw, 02–676, Poland and are available from the corresponding author upon request.
